The article "Sports Training Health Analysis Algorithm Based on Heart Rhythm Feature Extraction and Convolutional Neural Network" was retracted in 2023. Reasons: unreliable results or conclusions; concerns about the data; concerns about the peer review; concerns about the citations.

# Sports Training Health Analysis Algorithm Based on Heart Rhythm Feature Extraction and Convolutional Neural Network

**DOI:** 10.1155/2021/2946044

**Published:** 2021-08-30

**Authors:** Jing Li, Yunhang Lu, Ziyi Xiao

**Affiliations:** ^1^Sports Center, Xi'an Jiaotong University, Xi'an, Shaanxi 710049, China; ^2^Department of Physical Education, Kyungpook National University, Daegu 41566, Republic of Korea; ^3^Teaching and Research Office of College Physical Education, Yanching Institute of Technology, Langfang 065201, China

## Abstract

Intelligent sports equipment and software have emerged in the field of sports as a result of the advancement of information technology, allowing professional athletes to collect and visually display the movement and physical signs of the human body to aid in the planning of sports strategies. Intuitive data, on the other hand, cannot assist ordinary people who lack professional knowledge in exercising correctly. As a result, in the field of intelligent sports and health, effective use of collected exercise and physical sign data to analyze the user's personal physical condition and generate reasonable exercise suggestions has emerged as a research direction. In humans, the heart sound signal is a biological signal. It can help people detect and monitor heart health problems by analyzing the characteristics of heart sound signals. The goal of this paper is to use heart sound to identify and analyze athletes' training health. It provides a revolutionary health analysis algorithm based on heart rhythm feature extraction and convolutional neural networks, which is based on exercise training. It greatly improves the accuracy of the recognition and prediction of the athlete's training health status.

## 1. Introduction

The economic status of today's society is improving all the time, but fast-paced work and rising living costs have had a significant negative impact on people's health [1–3]. Young and middle-aged adults' adult physical fitness indexes dropped by an average of 0.5 percent. As a result, there are still flaws in people's physical health [4, 5], particularly among adults who are under a lot of work and life stress. Sports are an effective way to keep the human body healthy on a daily basis [6], and numerous studies have shown that using the right exercise methods and getting enough exercise can improve physical fitness and health in people of all ages.

As a part of the sports health market, sports fitness has also developed rapidly in recent years. According to estimates, the scale of China's online sports fitness market reached 174 billion yuan in 2019, and the number of users reached 195 million. The huge user scale brings a huge amount of information and data, which contains great value. At present, sports health applications [7–10] are more focused on data collection [11] and data visualization display [12–14] and lack further analysis and mining of user health data. Reasonable advice and help is the main direction of sports and health applications in the intelligent age.

In recent years, technologies such as the Internet of Things [15, 16], big data [17, 18], cloud computing [19, 20], and artificial intelligence [21–23] have gradually matured. The Internet of Things technology represented by 5G has promoted the in-depth development of the mobile Internet and provided an infrastructure for large-scale real-time user data acquisition. In order to improve resource utilization, cloud computing integrates storage and computing resources into a scalable and expandable resource pool, which has large-scale computing and storage capabilities. Customers can uniformly manage and schedule resource pools through the network, with great flexibility. Therefore, cloud computing has the advantages of reducing hardware costs, enhancing independent development capabilities, and improving resource utilization. Big data technology can quickly store and calculate massive amounts of data, provide enterprises with more accurate decision-making assistance, increase productivity, and reduce production costs. Artificial intelligence technologies such as deep learning and machine learning have aided the industry's evolution toward unmanned and intelligent operations, allowing customers to obtain more precise unmanned services, lower societal production costs, and increase service quality. Integrating technologies such as the Internet of Things, cloud computing, big data, and artificial intelligence to achieve a low-cost, intelligent, and precise sports health cloud platform can promote the development of the sports health industry and provide advanced technical assistance for improving the physical health of the people.

The goal of this paper is to look at the problem of sports health prediction [24–26] and recognition from the standpoint of heart sound periodic feature extraction methods and heart sound neural network structure design. To provide accurate services for athletes and promote the development of sports health and intelligence, a sports training health analysis algorithm based on heart rhythm feature extraction and convolutional neural network is proposed.

Following are the main innovations of this paper:

1. The proposed novel method can use the current mainstream classifier with the image and biological signal-based convolution neural network (CNN) and further combine CNN and heart sounds feature extraction method. It can be used for recognizing the heart sounds of the athletes training.
2. In this paper, heart sound convolutional neural network is designed to solve the problem of heart sound recognition and classification based on the extraction of heart sound periodic features. This paper studies the heart sound signal preprocessing, the feature extraction method, and the structure design of the heart sound neural network, starting from the mathematical definition and deducing the experimental method.

The rest of the article is organized as follows. In Section 2, background study and literature review are elaborated. The methodology is discussed in Section 3, followed by experimental setup and results in Section 4. Finally, Section 5 concludes the paper.

## 2. Background

Sports health services [27] include exercise advice, physical fitness monitoring, etc. Among them, exercise advice is also called exercise prescription. It was proposed by physiologist Kapović in the 1950s. Due to the difference in human physique, each person's suitable exercise method and amount of exercise vary. There are big differences. Just like the form of medical consultation, exercise advice is customized according to the user's own physical characteristics, forming the concept of exercise prescription. The traditional sports generation is a one-to-one method, which is limited by the scale of sports prescription experts and cannot meet large-scale needs. With the emergence of big data and artificial intelligence technology, especially the mature and unmanned artificial intelligence technology, intelligently generating exercise prescriptions and providing precise services for users has become a major direction of sports health services.

With the development of data information technology such as big data and machine learning [28, 29], using data algorithms to mine valuable information from large amounts of data has become a hot topic of data research [30, 31]. The sports health application, which collects a large number of users' sports and physical signs data, can use data information technology to dig out valuable information, so that the sports assistant service can be more intelligent and personalized.

Data analysis can assist people in comprehending the various types and structures of data, but such a superficial understanding of data is insufficient to perform the data's intended function. Data also assist humans in focusing on the information contained in data analysis, which is the true value of data. Such information can be classified as biological or nonbiological. Genomic data, microbiome data, personalized medicine data, and disease data are examples of biological type data, and this topic focuses on the types of data found in personalized medicine and disease data. It is well known that a certain biological signal data contains the physiological characteristics of the organism, and we can analyze the biological information from such biological signal data. Like the uniqueness of the organism, its biological signal also has certain uniqueness.

These data have become a treasure trove for many researchers. By studying the biological signals of the same organism, we can understand the differences between these data, so that we can draw some quantitative or regular conclusions. When we have data like the amount of lactic acid in the muscle at rest and the amount of lactic acid in the muscle at exercise, it can help us draw some accurate conclusions. It can be said that the development of data collection and analysis methods has helped us understand the laws of life more and more. There are also many biosignal data in humans, which are beneficial to the researchers studying the physiological structure of human beings and the pathologic causes of human beings.

In recent years, convolutional neural network (CNN) has emerged in the field of neural networks, especially in the field of image recognition, which has an unprecedented effect. In the classification and recognition of images, CNN has a wide range of application prospects. Not only that, but for medical images, it is also within the scope of CNN. At present, in the research on heart sound signals in academia, many researchers use deeper and more complex networks and more computing resources in pursuit of higher accuracy, and the methods used by these researchers to improve accuracy are of very high standard. Special consideration is seldom given to storage space and computing resources. The included platforms have limited computing power in real-world applications, such as hand-held heart sound filters, wearable life suits, and other tasks, due to production costs and actual market demand, and these platforms are all real time. Inspectors must be able to obtain test results quickly while keeping costs low, so these platforms must be able to process classification and recognition tasks quickly. As a result, in the engineering of heart sound classification and recognition, a neural network with fewer parameters and calculations is more feasible.

## 3. Methodology

### 3.1. Collection of Athletes' Heart Sounds

In the process of heart sound acquisition, attention should be paid to the following three aspects in the design of heart sound acquisition device.

First, ambient noise should be considered. This is a problem that will be encountered in all the processes of heart sound signal acquisition, which requires extra attention and efforts to reduce the impact of environmental noise.

Second, errors from the acquisition device and the operator's misoperation should be considered. This can be improved or avoided during the collection process, such as handling lightly and selecting sensors with better performance for the collector.

Third, other biological signals from the gatherers themselves should be considered. In the human body, there are other biological signals besides a heart sound, for example, lung sounds, so if the collector picks up heart sounds right after strenuous exercise, they will be different from the heart sounds that are picked up at rest.

Therefore, this section reviews the current situation of heart sound acquisition equipment and looks forward to more intelligent heart sound acquisition devices in the future from the composition to the specific structure. This is shown in Table 1.

### 3.2. Heart Sound Signal Preprocessing

#### 3.2.1. Heart Sound Resampling

The original heart sound signal is typically sampled at 22050 Hz. The sampling point is relatively large when compared to the signal's frequency. The difference between the two is an order of magnitude, so there is a lot of original sampling data. The frequency range of the heart sound signal is 101000 Hz, so there is a lot of original sampling data. It can be said that the majority of the data in these data are other irrelevant signals and may even be interference signals. Therefore, such a sampling rate increases the possibility of noise, and the huge amount of data also increases the signal. The time complexity and space complexity of processing will affect the speed of processing heart sound signals. So, it is necessary to resample the original heart sound signal. This section uses a sampling rate of 2000 Hz, and the sampling effect is shown in Figures 1(a) and 1(b).

#### 3.2.2. Wavelet Denoising

Because the heart sound signal is a biological signal with a low signal strength, it is easily disturbed by noise in signal collection or processing. If the noise in the signal is not removed, it will have a significant impact on the use of heart sound in disease diagnosis. As a result, the heart sound signal must be denoised. For example, the aforementioned heart sound signal collection device can recognize that current technology has yet to achieve zero noise for heart sound signal collection. Therefore, it is necessary not only to rely on hardware measures to solve the interference problem but also to have a specific signal filtering technology to participate in it, which lays a good foundation for various studies of heart sound signals.

The selection of wavelet basis function and the determination of the number of signal decomposition layers are two important aspects that affect the performance of wavelet denoising. If the selection of wavelet basis is not good, the whole performance will suffer loss.

Therefore, both the small heart sound signal and the noise signal are separated, if you choose too many levels of decomposition, but if you choose too few levels of decomposition, you filter out some of the useful signals. It is very important to choose the wave basis function or to determine the number of decomposition layers. The denoising process of heart sound signal using wavelet can be summarized as the following basic steps:

1. Select the wavelet basis function most suitable for heart sound signal.
2. Determine the number of decomposition layers *N*.
3. According to the decomposition level *N*, the heart sound signal is decomposed in *N* layers.
4. For the high-frequency coefficient of each layer obtained after decomposition, soft 1}7 value or hard 1}7 value is selected for quantitative processing.
5. If the effect is not good, return until the best effect is obtained.

#### 3.2.3. Hilbert Transform

Because the heart sound is a quasiperiodic signal and this paper is a periodic study of the heart sound signal, this section employs the envelope extraction method without indicating the heart sound's position. In fact, the height of the peak in the time domain for heart sounds contains the characteristics of the heart sound signal, which can be reflected in the heart sound signal's envelope.

In signal analysis tools, Hilbert transform is an important method. Hilbert transform is generally used to extract the phase information of the signal, calculate the envelope of the signal, and analyze the spectrum information of the signal. The definition of Hilbert transform is given below. Suppose there is a signal *x*(*t*), after Hilbert transformation, $\hat{x}\left(t\right)$ can be obtained from the following equation:

(1) $$\begin{array}{c} \hat{x}\left(t\right)=H\left(x\left(t\right)\right)\\ =\frac{1}{\pi }\int_{-\infty }^{\infty }\frac{x\left(\tau \right)}{t-\tau }d\tau =\frac{1}{\pi }\int_{-\infty }^{\infty }\frac{x\left(t-\tau \right)}{\tau }\\ =x\left(t\right)\times \frac{1}{\pi t}. \end{array}$$

It can be seen from equation (1) that the output signal is linearly related to the input signal divided by time. Just like the relationship between voltage and current, a filter is added in between. Therefore, this transformation can be turned into a filter, and the output response of the filter is set to *h*(*t*); then:

(2) $$\begin{array}{c} h\left(t\right)=\frac{1}{\pi t}. \end{array}$$

The above formula can be seen in the form of the signal in the time domain. But the Hilbert transform is mainly to analyze the frequency-domain relationship of the signal, so we need to know the frequency response *H*(*f*) of the Hilbert transform.

(3) $$\begin{array}{c} H\left(f\right)=-j\mathrm{sgn}\left(f\right)=\left\{\begin{array}{cc} -j, & f<0,\\ j, & f>0. \end{array}\right) \end{array}$$

Therefore, after the Hilbert transform of the signal *x*(*t*), the result in the frequency domain is the spectrum shift. The signal with positive frequency rotates 90° counterclockwise in the frequency domain, that is, the phase shift is reduced by 90°. The signal with negative frequency rotates 90° clockwise in the frequency domain, which increases the phase shift by 90°. Therefore, there is a difference of 180° between the positive frequency signal and the negative frequency signal. If the output signal is described as $\hat{x}\left(t\right)$ and the input signal is described as *x*(*t*), the envelope of the signal can be obtained. Therefore, if the envelope signal is set as *z*(*t*), the equation can be obtained:

(4) $$\begin{array}{c} z\left(t\right)=x\left(t\right)+\hat{x}\left(t\right). \end{array}$$

The original signal is shown in Figure 2.

The heart sound envelope obtained by the Hilbert transform method is shown in Figure 3.

The original signal is represented by a blue curve, and the envelope curve is represented by a red curve. In the Hilbert transform, an envelope curve of the same length of the signal can be obtained, that is, the envelope characteristic of the signal can be completely expressed.

### 3.3. Heart Sound Convolutional Neural Network

The architecture of the depth model can be determined by the total number of layers *n* and the number of structures in each stage {*a*_*i*_}. For example, *n*=3 and *a*_1_, *a*_2_, *a*_3_=4,3,2 indicate that the model has 3 stages, and the number of convolutional layers in the first, second, and third stages is 4, 3, and 2, respectively. Before deriving the formula, you need to define some required parameter symbols, which are the input spectrogram size *z*, the convolution kernel size *k*, and the minimum *c* value *t*. This paper requires that the *c* value of all layers is not less than the minimum *c* value *t*. As the receptive field of the convolutional layer continues to grow and the size of the convolution kernel in each convolutional layer remains unchanged, it can be seen that the *c* value of the last convolutional layer is the smallest. Therefore, it is equivalent to ensuring that the *c* value of the last layer in each convolutional layer is not less than *t*, which can be converted into a set of inequalities:

(5) $$\begin{array}{c} \frac{2^{l}k}{\sum_{i=1}^{l}2^{i-1}\left(k-1\right)a_{i}}\geq t,l=1,2,\cdots ,n, \end{array}$$

where 2^*l*^*k* is the size of the receptive field of the last layer of the convolutional layer ∑_*i*=1_^*l*^2^*i*−1^(*k* − 1)*a*_*i*_ of the *l*-th layer. The receptive field at the top of the convolutional layer should be smaller than the area of one heart sound cycle. That is, the formula is expressed as follows:

(6) $$\begin{array}{c} \sum_{i=1}^{l}2^{i-1}\left(k-1\right)a_{i}\leq z. \end{array}$$

The objective function can be expressed in the form of the total number of maximum pooling layers, and its final equation is

(7) $$\begin{array}{c} \underset{n,\left\{a_{i}\right\}}{\max}\sum_{i}^{n}a_{i},\\ \sum_{i=1}^{l}2^{i-1}a_{i}\leq \frac{2^{l}k}{t\left(k-1\right)},\;l=1,2,\ldots ,n,\\ \sum_{i}2^{i-1}a_{i}\leq \frac{z}{k-1}. \end{array}$$

The model of the heart sound convolutional neural network designed in this paper is shown in Figure 4.

## 4. Experiments and Results

### 4.1. Experimental Setup

This experiment uses the PyCharm compiler and the TensorFlow deep learning framework in the Windows environment and uses the constructed heart sound convolutional neural network to predict and recognize the athlete's training health status. Using a small batch learning method, Adam optimizer, the learning rate is 0.0001, and a total of 1000 iterations are performed.

### 4.2. Datasets

This article uses the PhysioNet/CinC Challenge 2016 database. All recordings have been resampled to 2000 Hz, and the duration of the recordings ranges from 5 seconds to more than 120 seconds. The ultimate goal of this study is to divide them into two types of normal and abnormal heart sounds. The training set consists of five data folders (A to E), containing a total of 3240 heart sound recordings, and the test set contains 301 heart sound recordings. In this study, by extracting 5 cardiac cycles as the time length of a spectrogram, a total of 28,000 training samples are obtained. There are 4800 test samples.

### 4.3. Evaluation Index

Relative error (RE) takes the actual value as the reference value and judges by comparing the relative difference between the predicted result of the target data and the actual value. We usually express it as a percentage. The smaller the value of the relative error is, the closer the prediction result is to the actual value. In other words, the better the prediction effect of the constructed model. Generally speaking, the relative error can better reflect whether the prediction result is credible. The relative error expression is as follows:

(8) $$\begin{array}{c} \mathrm{RE}=\frac{y_{i}-y_{i}^{\prime }}{y_{i}}\times 100\%. \end{array}$$

### 4.4. Experimental Results

On the basis of the designed basic heart sound neural network structure, the complexity of the model is optimized by changing the number of convolutional layers, and the model is verified experimentally; the parameters of the heart sound classification model, training time, and accuracy of training are shown in Table 2.

Some conclusions can be drawn from Table 2. When there is only one convolutional layer, the amount of model parameters is huge, important features cannot be accurately obtained, and the training time is long; when there are three convolutional layers in the model, the training time is short and the number of parameters is small, but the accuracy rate is reduced, and in the case of two convolutional layers, the training time is acceptable and the accuracy is the highest.

This paper realizes the design of adapting to the heart sound signal by improving the structure. In order to illustrate the effectiveness of the model designed by the method proposed in this paper, the heart sound challenge database dataset is used as the data source. The fixed number of training steps is 10,000 steps. We change the batch_size of the model in this section to different values for comparative analysis. The training process is shown in Figure 5.

It can be clearly seen from Figure 5 that when the batch_size is 32, the optimal effect can be obtained. However, because the training of 10,000 steps is too small for the general CNN, the following fixes the batch_size size and changes the number of trainings in order to obtain the best model.

### 4.5. Ablation Research

We verify the influence of the custom parameter learning rate on the performance of the proposed algorithm. We set up a set of ablation experiments and selected 4 different learning rates for simulation experiments. The experimental results are shown in Table 3.

It can be seen from Table 3 that if the learning rate is reduced, the performance is increased as a whole, until it reaches the highest value at 0.0001. Secondly, after the learning rate is reduced again, the performance decreases. Therefore, this proves that the learning rate setting of the proposed algorithm is correct.

### 4.6. Limitation

Although the model based on heart rhythm feature extraction and convolutional neural network proposed in this paper has achieved effective results, the heart sound signal is a kind of time series data, which involves the dependence of long-distance information. There are certain limitations in feature extraction. In the next study, we will investigate the effectiveness of recurrent neural networks in extracting features of heart sound signals.

## 5. Conclusion

In this paper, we believe that the effective use of collected exercise and physical sign data to analyze the user's personal physique and generate reasonable exercise suggestions has become the research direction in the field of intelligent exercise and health. The heart sound signal is a biological signal that exists in humans. By analyzing the characteristics of heart sound signals, it can help people detect and monitor heart health problems. The purpose of this paper is to identify and analyze the training health of athletes by heart sound. It uses the current mainstream convolutional neural network (CNN) on images and biosignals in the classifier and combines CNN with heart sound feature extraction methods to propose a novel method based on sports training health analysis algorithm based on heart rhythm feature extraction and convolutional neural network. It greatly improves the accuracy of the recognition and prediction of the athlete's training health status.

## Figures and Tables

**Figure 1:** Signal sampling.

**Figure 2:** Waveform of normal heart sound in time domain.

**Figure 3:** The original signal and the heart sound signal after obtaining the envelope.

**Figure 4:** Heart sound convolutional neural network model.

**Figure 5:** Comparison results of different batch_size. (a) Batch_size = 8, steps = 1000. (b) Batch_size = 16, steps = 1000. (c) Batch_size = 32, steps = 1000.

**Table 1:** Heart sound collection equipment.

Equipment name	Legend
Electronic stethoscope	
Bluetooth stethoscope	
Wearable heart sound stethoscope	
Doppler stethoscope	
Smart stethoscope	

**Table 2:** Classification effects of models with different numbers of convolutional layers on heart sounds.

Convolution kernel size	Parameters	Training time (m)	Accuracy
(3, 3, 3)	21584525	37	0.9412
(7, 7, 3)	21325455	36	0.8852
(11, 11, 3)	22147223	46	0.8156

**Table 3:** Results of ablation studies.

Learning rate	Accuracy
0.01	0.9388
0.001	0.9401
**0.0001**	**0.9412**
0.00001	0.9403

The bold values represent the best performance of the adopted method.

## Data Availability

The data used to support the findings of this study are included within the article.
